The article "The Effect of Suppression Taurine on Relocation and Epithelial-Mesenchymal Transition in Mankind Lung Cancer Cells" was retracted in 2023. Reasons: signs of a paper mill; suspected computer-generated content; unreliable results or conclusions; concerns about the data.

# The Effect of Suppression Taurine on Relocation and Epithelial-Mesenchymal Transition in Mankind Lung Cancer Cells

**DOI:** 10.1155/2021/6656080

**Published:** 2021-04-14

**Authors:** Yongyan Deng, Hongjin Li, Yujiao Tang

**Affiliations:** ^1^Changchun Sci-Tech University, Changchun 130-600, China; ^2^Jilin Sino-ROK Institute of Animal Science, Changchun 130-600, China

## Abstract

**Aim:**

Taurine is believed to have antioxidant properties and has been implicated in the treatment of neurodegenerative disease, atherosclerosis, coronary heart disease, and prostate cancer. This research focused on taurine inhibition effects of expression related to migration and epithelial-mesenchymal transition- (EMT-) A549 study on related genes of human being non-small-cell lung cancer.

**Methods:**

MTT assays assessed cell viability and a Radius^TM^ assay showed that taurine also inhibited the lung cancer cell migration. Using RT-PCR and Western blot, the migration and EMT markers were identified and evaluated.

**Results:**

We found that taurine significantly decreased the expression of migration markers matrix metallopeptidase 9 (MMP-9) and vascular endothelial growth factor (VEGF). In contrast, TIMP metallopeptidase inhibitor 1 (TIMP-1) and TIMP metallopeptidase inhibitor 2 (TIMP-2) expressions were increased with taurine treatment. In addition, we found an association between taurine treatment and the expression of EMT markers. The expression of epithelial marker E-cadherin and the mesenchymal marker N-cadherin TWIST-1 was decreased, but the expression of zinc finger protein SNAIL-1 and E-zinc finger homeobox 1 (ZEB-1) was increased.

**Conclusion:**

Taken together, our study strongly suggests the therapeutic significance of taurine, which possesses antimigration activity and induces EMT markers expression in lung cancer cells.

## 1. Introduction

Worldwide, lung cancer has the highest incidence and mortality rate among all malignancies-related deaths mostly in men and smoking is known to be the primary cause [1–3]. Current studies have shown that the possibility of lung cancer in smokers is higher than 10–20 times than that in nonsmokers in the long term [2]. Although there has been significant progress over the last decade in the early detection and combined treatment of lung cancer, the incidence of five-year survival rate is still below 20% for those who have an advanced stage of lung cancer (cancer statistics, WHO). The initial step in tumor metastasis is the invasion of cancer cell. The invasion of this cancer cell takes place in surrounding tissue and vasculature. The protrusive activity of the cell membrane and the attachment to the extracellular matrix induce chemotic migration which is required for the invasion [4]. Tumor cell can secrete vascular endothelial growth factor (VEGF) which stimulates migration and proliferation and prolongs the survival of quiescent endothelial cells by activating transduction pathways [5, 6]. Matrix metalloproteinases (MMPs) belong to the endopeptidases family which is significant in cancer metastasis. MMP-2 and MMP-9 originally belong to the gelatinase protein family. Overexpression of MMP-2 and MMP-9 leads to tumor aggressiveness and poor prognosis, thereby degrading type IV collagen comprising basement membranes [7]. In addition, matrix metalloproteinases (TIMPs) tissue inhibitors regulate the active MMPs tightly [8]. TIMP-1–4 play a necessary role in the regulation of MMP factors [9].

The article "The Effect of Suppression Taurine on Relocation and Epithelial-Mesenchymal Transition in Mankind Lung Cancer Cells" was retracted in 2023. Reasons: signs of a paper mill; suspected computer-generated content; unreliable results or conclusions; concerns about the data.

Epithelial-mesenchymal transition (EMT) results in carcinoma cells with migratory and invasive properties [10]. After the EMT, loss of epithelial polarity of tumor cells, reduced adhesion between cells, and motor ability of tumor cells increased, resulting in the fact that the invasion of tumor cells significantly enhanced. Migration is inhibited in pre-EMT cells due to tight cell-to-cell junctions. Studies show that the movement of cells via tissue by increasing invasion of EMT positively correlates with migration. Post-EMT cells have higher migratory abilities, resulting in transcription of E-cadherin [11]. The epithelial biomarker E-cadherin is a tumor suppressor which is regulated by the Slug, SNAIL, and TWIST transcription factors. The expression of pluripotent genes is enhanced by R-cadherin which is a transmembrane calcium-dependent adhesion molecule [12]. N-cadherin is an EMT-regulated gene and a cell adhesion molecule with metastatic effects on cancer cells, which promotes embryonic left-right asymmetry. SNAIL regulates EMT during embryonic progression by suppressing the adhesion of E-cadherin. E-cadherin promotes the expression of the embryonic transcription factor TWIST by downregulating [13]. ZEB-1 induces oncogenic properties in invasive and metastatic lung cancer cells, which induces EMT [14]. The study found that EMT-related markers are closely related to pathological staging and prognosis in patients with lung cancer.

Taurine is widely distributed in animal tissues and marine animals. It is a byproduct of the sulfurous amino acids cysteine and methionine and acts as a lipid/membrane stabilizer in the body. The researches have shown that taurine has antioxidation, anti-inflammatory, and anticancer, improves the endocrine status, and enhances human immune function [15–18]. Taurine supports various biological functions like neurological development and water and mineral level regulation in the blood. It is especially used in infant formulas and even as total parenteral nutrition worldwide. Dietary sources supply the majority of the taurine for physiological and nutritional requirements and the small intestine absorbs this dietary taurine. Therefore, a higher concentration of taurine is observed in the small intestine [4]. However, researches on the antilung cancer properties of taurine are lacking. Therefore, we aim to find out the effect of taurine on A549 lung cancer cells, specifically in terms of the expression of migration and EMT-related genes.

The article "The Effect of Suppression Taurine on Relocation and Epithelial-Mesenchymal Transition in Mankind Lung Cancer Cells" was retracted in 2023. Reasons: signs of a paper mill; suspected computer-generated content; unreliable results or conclusions; concerns about the data.

## 2. Materials and Method

### 2.1. Materials

We purchased the human lung cancer cell line A549 from the Korean Cell Line Bank (Seoul, Korea; KCLB number: 10185). The Roswell Park Memorial Institute- (RPMI-) 1640 medium, fetal bovine serum (FBS), penicillin/streptomycin (P/S), and phosphate-buffered saline (PBS) for cell culture were all from Invitrogen (Carlsbad, CA, USA). Tris HCL buffer, sodium dodecyl sulfate, tris(hydroxymethyl)aminomethane, 2-mercaptoethanol, glycine, MTT formazan, sodium chloride solution, potassium chloride, potassium chloride, ethylenediaminetetraacetic acid disodium salt dihydrate, potassium phosphate monobasic, brilliant blue *G*, ammonium nickel sulfate hexahydrate, dimethyl sulfoxide, and 3,3-diaminobenzidine were purchased from Aladdin (Shanghai, China). N,N,N′,N′-Tetramethylethylenediamine, chloroform, 5% nonfat-dried milk, and taurine were purchased from Sigma-Aldrich (St. Louis, Missouri, USA). WesternBright Sirius HRP substrate was purchased from Advansta (Menlo Park, California, USA). 10X TBS with Tween 20 was purchased from Biosesang (Seongnam-si, Gyeonggi-do, Korea). 10% ammonium persulfate solution was from (Metropolitan City, Daejeon, Korea). TRIzol™ Reagent and the lane the labeling sample were bought from Thermo Scientific (Waltham, MA, USA). The other reagents used in this experiment are of the highest quality.

### 2.2. Cell Culture

The human lung cancer cell line A549 was cultured in RPMI 1640 medium with 10% of FBS in a 5% of CO_2_ atmosphere at 37°C. The MTT assay used 1.0 × 10^3^–1.0 × 10^4^ cells/well, and 3.5 × 10^5^ cells/well were planted in a 12/24 well culture dish. After 24 h, 0, 62.5, 125, 500, and 1000 *μ*M of taurine were added to the cells for 24 h for cell migration and invasion test, mRNA expression assay, and Western blot assay.

### 2.3. Cell Survival and Growth Assay

The human lung cancer cell line A549 cells for culture were used, and the MTT assay was used to study cell survival and growth assay. Collect the cells in the logarithmic growth phase, adjust the concentration of the cell suspension, add 100 *μ*L to each well, and plate to adjust the density of the cells to be tested to 1000–10000 wells. Incubate with 5% CO_2_ at 37°C until the cell monolayer covers the bottom of the well (96-well flat bottom plate), add concentration gradient drugs, administer and culture after 24 hours, and set up a control group. After incubating for 24–48 hours, add 10 Ul MTT solution to each well and spend 4 hours to incubate. Aspirate the supernatant carefully, and at the same time, add 100 *μ*L dimethyl sulfoxide to each well. And in order to completely dissolve the crystal, shake it on a shaker at low speed for 10 minutes. Measure the absorbance value at 570 nm of the enzyme-linked immunoassay (Anthos 2010, Salzburg, Austria) [19].

The article "The Effect of Suppression Taurine on Relocation and Epithelial-Mesenchymal Transition in Mankind Lung Cancer Cells" was retracted in 2023. Reasons: signs of a paper mill; suspected computer-generated content; unreliable results or conclusions; concerns about the data.

### 2.4. Cell Migration and Invasion Test

The Radius^TM^ 24-well cell migration assay (Cell Biolabs, Inc., San Diego, CA, USA) was used to study cell migration and invasion [20]. To determine cell migration, we put the 0.5 mL of solution A (gel pretreatment) on every place. The dish was allowed to react at 25°C for 30 min. Solution A was then discarded, and each well was washed with 0.5 mL of solution B (clean solution) placed into every place. The A549 cells were inoculated after they were put into the culture medium (RPMI + 10% FBS) at 3.5 × 10^5^ cell/mL. The A549 cells were cultured for 24 hours at cell incubator. After 24 hours, pour out the culture medium and wash them with 0.5 mL solution B three times. In the process, be gentle. Finally, the fresh culture medium was added after cleaning once again with medium. 1 mL of taurine and complete medium was added after the final washing and pictures were taken at 0, 6, 12, and 24 hours. In order to determine the difference between migration and invasion gaps, the images are of the same size and collected under gap closure which are analyzed by software (CellProfiler^TM^, Broad Institute, Cambridge, MA, USA).

### 2.5. mRNA Expression Analysis

TRIzol was used to extract total cellular RNA from harvest A549 cells. TRIzol preserves RNA integrity in the lysate or homogenate of the sample. After removing the water layer, nucleic acid and protein in the sample can be decreased successively in the form of rain. Ethanol precipitation can precipitate DNA in the middle layer [21]. The PCR amplification conditions are as follows: incubate at 95°C for 15 minutes, then denature at 95°C for 40 cycles of 30 s, and anneal in the transition temperature range of 58–62°C; each cycle increases by 0.5°C and extends at 72°C for 30 s. For each sample, the expression level of GAPDH was normalized to the expression level of the gene and presented relative mRNA levels. The primer sequence was shown in Table 1.

The article "The Effect of Suppression Taurine on Relocation and Epithelial-Mesenchymal Transition in Mankind Lung Cancer Cells" was retracted in 2023. Reasons: signs of a paper mill; suspected computer-generated content; unreliable results or conclusions; concerns about the data.

### 2.6. Extraction and Determination of Total Cell Protein

After discarding the nutrient solution, put the bottle upside-down on blotting paper, and allow the blotting paper to soak up the remaining nutrient solution. Add 3 mL of PBS buffer solution (0.01 M pH7.2 ～ 7.3) precooled at 4°C into cells' prebottle. Flat on the table and take a minute to slightly wobble to wash the cells, and then remove the liquor. Duplicate the above-mentioned experimental manipulation twice and wash the cells thrice to wipe out nutrient solution. Remove the PBS solution and posit culture bottle upon the ice. Put reagents according to the standard of 1 mL lysis buffer into 10 *μ*L PMSF (100 mM), and rock the culture flask on ice. Add 400 *μ*L of PMSF-containing lysate into each flask of cells, and spend 30 minutes on ice for lysis. The culture flask needs to be shaken back and forth frequently so that the cells can be fully lysed. When the lysis is complete, the cells are scraped on the side of the flask with a neat scraper (quickly); use 1.5 mL centrifuge tube to hold cell debris and lysate and centrifuge at 4°C at 12000 rpm 5 min, and store at −20°. Use BAS to establish a standard curve to determine the protein concentration.

### 2.7. SDS-PAGE Polyacrylamide Electrophoresis

Prepare SDS separation glue (*T* = 7.5%), pour into 10 cm × 10 cm glass plates, seal off the water, after the glue polymerizes, discard the water, and inject SDS concentrated glue (*T* = 4%). Add protein sample and prestained standard protein with a molecular weight of 26 ∼ 118kd, 20 *μ*g/well, 20 *μ*l/well. After electrophoresis, adjust 80 V, 1 h, to 100 V, 4 h. Stop electrophoresis until the front of bromophenol blue is 0.5 cm away from the lower edge of the glass plate.

### 2.8. Semidry Electrophoresis Transfer

After the electrophoresis, remove the gel and immediately immerse the gel in the cathode buffer (25 mM Tris, 40 mM Gly, 0.1% SDS, pH7.6). Shake for 20 min, place a PVDF membrane equal to the size of the gel (pore size 0.45 mm), and slowly immerse the PVDF membrane in 100% methanol at a 45° angle for 15 seconds until the PVDF membrane becomes uniform and transparent and sinks. Take out the membrane and immerse it in deionized water for 2 minutes, and then immerse it in anode buffer (25 mM Tris, 15% methanol, pH 10.4) for 5 minutes. Take 3 sheets of ordinary filter paper of the size of the membrane and immerse them in the anode buffer until they are saturated, and then take 3 sheets of filter paper and immerse them in the cathode buffer until they are saturated. Clamp the sandwich on the anode plate of the semidry transfer instrument. The order from the anode plate to the cathode plate is 3 sheets of filter paper immersed in anode buffer, PVDF membrane, and gel and 3 sheets of filter paper immersed in cathode buffer. Cover the negative electrode plate and perform the electrophoretic transfer. Electric transfer parameters are as follows: 4°C, 1.0 mA/cm2 film, 1 h.

The article "The Effect of Suppression Taurine on Relocation and Epithelial-Mesenchymal Transition in Mankind Lung Cancer Cells" was retracted in 2023. Reasons: signs of a paper mill; suspected computer-generated content; unreliable results or conclusions; concerns about the data.

### 2.9. Western Blot

After the electroporation, the PVDF membrane was immediately immersed in the dilution buffer (Tris 2.4 g, NaCl 8.0 g, dissolved in 1,000 mL, adjusted to pH 7.6, and 0.05% Tween-20 was added immediately before use) and washed for 5 minutes, according to the molecular weight of marker to predict the location, cut a small membrane on a 0.45 mm PVDF membrane, place it in an incubator filled with blocking buffer (2.0 g bovine serum albumin dissolved in 100 mL dilution buffer), and shake at room temperature. Incubate for 1 hour, wash with dilution buffer 3 times × 5 min, and place the small membrane in the working solution of primary antibodies. In the incubation box with shaking at room temperature as above, place the small membrane in the incubation box containing the secondary antibody working solution in the incubation box with shaking at room temperature as above. Under low light, place the membrane in an incubation box containing a chemiluminescence substrate solution (prepared enzyme substrate and enhanced luminescence agent in a 1 : 1 volume ratio according to the product instructions before use). After shaking for 5 minutes, take it out and place it in a transparent and then in a dark room; the front side is close to the X-film and exposed for 20 s in the cassette. The X-film is washed with an automatic roll film processor to obtain the Western blotting pattern.

Primary antibody, VEGF, MMP-9, TIMP-1, and TIMP-2, was used with a dilution ratio of 1 : 2000 from Santa Cruz Biotechnology. The ZEB1, TWIST, E-cadherin, N-cadherin, actin, and SNAIL were purchased from Cell Signaling Technology with a dilution ratio of 1 : 3500. Used secondary antibodies, goat anti-rabbit, and goat anti-mouse (1 : 5000) were from Santa Cruz Biotechnology.

All of the data of this study were statistically analyzed by SAS statistical software (SAS Institute, Cary, NC, USA). To determine the treatment activity, one-way analysis of variance (ANOVA) was used.

## 3. Result

### 3.1. Human Lung Cancer Cell Viability Is Affected by Taurine

The cell survival and growth activity of taurine on lung cancer cells were evaluated by MTT assay. We found that the lung cancer cells die in a dose-dependent manner at a concentration of 250–1000 *μ*M (Figure 1). We would like to study the effect of a low concentration of taurine on lung cancer cells. Hence, 62.5–500 *μ*M was selected for the antilung cancer experiment. Therefore, 62.5–500 *μ*M was selected for further experiments.

The article "The Effect of Suppression Taurine on Relocation and Epithelial-Mesenchymal Transition in Mankind Lung Cancer Cells" was retracted in 2023. Reasons: signs of a paper mill; suspected computer-generated content; unreliable results or conclusions; concerns about the data.

It took 24 and 48 hours to incubate lung cancer cells with various concentrations of taurine and after 4 hours of MTT, 100 *μ*L of isopropanol was added to dissolve the formazan crystals. Each value is expressed as the mean ± SEM. ^*∗*^Significant difference from control group shown at *p* < 0.05 by Dunnett's multiple range test.

### 3.2. The Migration of Human Lung Cancer Cells Is Affected by Taurine

The Radius^TM^ 24-well plate was used for the gap closure assay, with the purpose of discovering the migration effect of taurine on lung cancer cells. Capture images in a smaller size. We have determined the narrowing of the gap according to the indicated times (0, 6, 12, and 18 h) to compare the variation in migratory gaps. As seen in Figure 2, after 18 h, the gap was minimized to 90.33% in the control group and cell motility reduced to 59.00% for taurine compared to the control group.

In the presence or absence of different concentrations of taurine, growth is allowed for a specified time. The cell coverage gap is fathomed by CellProfiler. The average of three independent experiments was performed in triplicate by gap representation. Each value is expressed as the mean ± SEM. ^*∗*^Significant difference from control group shown at *p* < 0.05 by Dunnett's multiple range test.

### 3.3. Migration and EMT-Related Gene Expression Are Affected by Taurine

We treated taurine in A549 cells for 24 h and performed reverse-transcription- (RT-) PCR. We investigated the angiogenesis promoting factor mRNA expression (Figure 3). VEGF expression was significantly decreased which indicated that the taurine suppressed migration in A549 human lung cancer cell. In additon, MMP-9 expression is dramatically reduced under the action of taurine. MMP-9 naturally occurring inhibitors such as TIMP-1 and TIMP-2 mRNA expression levels were dramatically increased for taurine in A549 cells. Then, we look for expression by Western blot standards of VEGF, MMP-9, TIMP-1, and TIMP-2. As shown in Figure 4, the expression of VEGF and MMP-9 was significantly decreased following taurine treatment, while standards of the MMP-9 inhibitors TIMP-1 and TIMP-2 were significantly enhanced. Our data show that taurine reduced the migration capability in A549 human lung cancer cells, adjusting the expression of TIMP-1 and TIMP-2.

It took 24 hours to treat the cells with various concentrations of taurine. (A) After waiting for 24 hours, harvest cells and isolate total RNA. Measure the gene expression level of genes related to migration (VEGF, MMP-9, TIMP-1, and TIMP-2) by RT-PCR (A). We standardize the mRNA levels of the analyzed genes in each sample according to the level of GAPDH (B). ^*∗*^Dunnett's multiple range test showed a dramatic difference from the control group at *p* < 0.05.

The article "The Effect of Suppression Taurine on Relocation and Epithelial-Mesenchymal Transition in Mankind Lung Cancer Cells" was retracted in 2023. Reasons: signs of a paper mill; suspected computer-generated content; unreliable results or conclusions; concerns about the data.

### 3.4. Influence of Downstream Gene Expression of EMT Is Affected by Taurine

Then, we analyzed the downstream signal of EMT, including E-cadherin, N-cadherin, TWIST-1, SNAIL-1, and ZEB-1. The indication standards of E-cadherin, N-cadherin, TWIST-1, SNAIL-1, and ZEB-1 were investigated using RT-PCR and Western blot. We found that taurine-induced E-cadherin expression improved, thereby reducing the expression level of N-cadherin TWIST-1, SNAIL-1, and ZEB-1 significantly in dose-dependent manners (Figures 5 and 6).

It took 24 hours to treat the cells with various concentrations of taurine. After waiting for 24 hours, harvest cells and isolate total RNA. The gene expression level of genes related to migration (N-cadherin, E-cadherin, TWIST-1, SNAIL-1, and ZEB-1) were measured by RT-PCR (A). We standardize the mRNA levels of the analyzed genes in each sample according to the level of GAPDH (B). ^*∗*^Dunnett's multiple range test showed a dramatic difference from the control group at *p* < 0.05.

## 4. Discussion

More and more reports show that taurine is used in food and beverage because of its high health care effect. Moreover, it has a high development prospect. Recent researches have indicated that taurine shows antiproliferative and antineoplastic properties in various cancer cells [22–24]. During the occurrence and development of cancer, cell growth regulation plays an important role in regulating its differentiation and apoptosis. Various stimuli, including chemotherapeutic agents and radiation, can activate apoptosis. It is a process where cell death is programmed genetically. Chromatin condensation, cell shrinkage, and nuclear fragmentation are common morphological features [25]. Various *in vivo* and *in vitro* researches have disclosed that many natural product agents can lead to this genetically programmed death in different types of cancer cells, referred to as apoptosis [26]. For this reason, taurine was estimated for its anticancer properties using an MTT assay. The data show the taurine-induced apoptosis in lung cancer. It followed a dose-dependent mannerism (Figure 1). Relevant concentration was selected for subsequent analysis.

EMT is interrelated to migration. Migration is influenced by cell-cell adhesion, with migration rates varying for cells with different cell-cell adhesion properties [27]. Cancer metastasis is influenced by cellular motility and migration [28]. In this study, we performed an *in vitro* model, Radius^TM^ 24-well cell migration assay, to find out the effect of taurine on lung cancer cell, A549. We carried out cell migration and invasion experiments with the Boyden chamber. The influence of taurine on lung cancer cell migration is reflected more clearly and accurately. Later, after 24 hours of inoculation, 90% of the bottom area of the cell culture plate was reached, and the gel was removed. In normal cell culture, the A549 cells were evenly distributed around the circle. When the special substance in the bottom circular area is removed, the cells will grow into a circle [29]. A549 cells were treated with and without taurine, and the migratory potential was determined by performing a gap closure assay. Taurine significantly repressed the migration of human lung cancer cells, A549 at various time points.

The article "The Effect of Suppression Taurine on Relocation and Epithelial-Mesenchymal Transition in Mankind Lung Cancer Cells" was retracted in 2023. Reasons: signs of a paper mill; suspected computer-generated content; unreliable results or conclusions; concerns about the data.

Metastasis occurs through a metastatic cascade which includes some series of steps [30]. VEGF is associated with metastasis expansion [31, 32]. VEGF can be responsible for angiogenesis and even poor prognosis in some old tumors [33]. We therefore determined the fact whether taurine inhibits VEGF or causes cell motility in lung cancer cells. Based on our experiments, we demonstrated that VEGF is suppressed by taurine in lung cancer cells.

MMPs are key factors for the remodeling of extracellular matrix which is associated with tumor development [34]. MMP-2 and MMP-9 are known to take part in essential acts Ectopic infiltration, implantation, adhesion, and neovascularization of various tumors [35]. Western spot analysis and RT-PCR of VEGF, MMP-2, MMP-9, TIMP-1, and TIMP-2 were conducted. We demonstrated that the expression of MMP-9 and VEGF is inhibited by taurine. However, we did not witness difference that taurine affects MMP-2 protein levels in A549 cells (data not shown).

There have been several previous studies reporting that MMP-9 and its particular suppressors, TIMPs, are firmly associated with pathological and physiological processes involving the degradation and ECM accumulation [35, 36]. Except for neutrophils, the secretion of TIMP-1 and TIMP-2 was positively and inversely proportional to MMP-9. The utterance of MMP-9 was high and the secretion of TIMP-1 and TIMP-2 decreased [37]. Interestingly, TIMP-1 has been found to be not only independently localized but also colocalized in neutrophil organelles [38]. Accordingly, we examined the mRNA standards of TIMP-1 and TIMP-2 and showed that the expression of TIMP-1 and TIMP-2 improved with the increase of taurine concentration.

To confirm these results, the expression level of VEGF is detected by RT-PCR and Western blot, MMP-9, TIMP-1, and TIMP-2. In Figures 3 and 4, the expression of VEGF and MMP-9 significantly decreased the following taurine treatment, while standards of the MMP-9 inhibitors TIMP-1 and TIMP-2 significantly increased.

The article "The Effect of Suppression Taurine on Relocation and Epithelial-Mesenchymal Transition in Mankind Lung Cancer Cells" was retracted in 2023. Reasons: signs of a paper mill; suspected computer-generated content; unreliable results or conclusions; concerns about the data.

EMT is known to act in embryonic development. Cells migrate to specific intents in the embryo due to mesenchymal attribution [39], where they undergo differentiation. To figure out the part of EMT in migration, we have exactly analyzed the utterance of some EMT markers using RT-PCR and Western blot, such as E-cadherin, N-cadherin, ZEB-1, TWIST-1, and SNAIL-1. In this context, E-cadherin is an important indicator of migration and invasion abilities. ZEB-1 and SNAIL-1 are the primary transcriptional factors for E-cadherin expression [38]. ZEB-1 enhances migration by upregulating E-cadherin. ZEB-1 may be associated with tumor grade in adenocarcinomas, regulating lymphatic and distant lung squamous cell carcinomas. SNAIL is essential for cell migration; it is a strong suppresser of E-cadherin and also a major EMT inducer [40]. Our consequences indicate that taurine prevails the downregulation of ZEB-1 and SNAIL-1 expression in a dose-dependent manner. N-cadherin and TWIST-1 are known to be important biomarkers for diagnosing lung cancer. N-cadherin is a transmembrane glycoprotein that promotes aggressive behaviors in the A549 cell line, such as invasion and migration, while TWIST-1 is a transcriptional catalyst of N-cadherin [40]. TWIST-1 promotes incursion in lung cancer cells and the downregulation of TWIST-1 in lung cancer cells drives the repression of N-cadherin. We found dose-dependent reductions in the expression of N-cadherin as well as TWIST-1 in cancer cells treated with taurine.

## 5. Conclusion

In summary, this research found that taurine has certain acting on inhibiting A549 human lung cancer cells; and it induces apoptosis, suppressing migration and altering the expression of migration-related and EMT-related proteins VEGF, MMP-9, TIMP-1, TIMP-2, N-cadherin, E-cadherin, TWIST-1, SNAIL-1, and ZEB-1. These data can serve as a reference for clinical development and drug development. However, this study was only carried out at the cell level. We will further study the anticancer effect of taurine in mouse lung cancer model.

## Figures and Tables

**Figure 1:** Analysis of cell viability of taurine on A549 cells.

**Figure 2:** The influence of taurine on the ability of intercellular space closure in A549 cells.

**Figure 3:** Effects of A549 cells migration-related genes through taurine.

**Figure 4:** Protein expression of migration-related genes in Western. (a) Normalize the expression of VEGF, MMP-9, TIMP-1, and TIMP-2 through *β*-actin. (b) ^*∗*^Significant difference from control group shown at *p* < 0.05 by Dunnett's multiple range test.

The article "The Effect of Suppression Taurine on Relocation and Epithelial-Mesenchymal Transition in Mankind Lung Cancer Cells" was retracted in 2023. Reasons: signs of a paper mill; suspected computer-generated content; unreliable results or conclusions; concerns about the data.

**Figure 5:** Influence of EMT-related genes in A549 cells affected by taurine.

**Figure 6:** Protein expression of EMT-related genes in Western. (a) Expression of N-cadherin, E-cadherin, TWIST-1, SNAIL-1, and ZEB-1 (b) ^*∗*^Dunnett's multiple range test showed a dramatic difference from the control group at *p* < 0.05.

**Table 1:** Primers.

Target gene	Primer sequence
VEGF	Forward 5′-GGG GCA GAA TCA TCA CGA AG-3′ Reverse 5′-TTT CTC CGC TCTGAG CAA GG-3′
MMP-9	Forward 5′-CGA CGT CTT CCA GTA CCG AG-3′ Reverse 5′-GTT GGT CCC AGT GGG GAT TT-3′
TIMP-2	Forward 5′-CAG CTT TGC TTT ATC CGG GC-3′ Reverse 5′-ATG CTT AGC TGG CGT CAC AT-3′
TIMP-1	Forward 5′-CAA GAT GAC CAA GAT GTA TAA AGG-3′ Reverse 5′-AAC AGT GTA GGT CTT GGT GAA G-3′
GAPDH	Forward 5′- CCA TGG GGA AGG TGA AGG TC-3′ Reverse 5′-AAA TGA GCC CCA GCC TTC TC -3′
N-cadherin	Forward 5′- ACC TCA AGA GGC AGA GAC TT-3′ Reverse 5′-CAG AGC AGG ATG GCA ATG AT -3′
E-cadherin	Forward 5′- TTG CGG AAG TCA GTT CAG A-3′ Reverse 5′-CGG GTG TCG AGG GAA AAA TA -3′
TWIST	Forward 5′-GCA TTC TCA AGA GGT CGT GC -3′ Reverse 5′-ATG GTT TTG CAG GCC AGT TTG -3′
SNAIL	Forward 5′-CCA ATG CTC ATC TGG GAC TC -3′ Reverse 5′-TTC GGA TGT GCA TCT TGA GG -3′
ZEB1	Forward 5′-TGG GAG GAT GAC ACA GGA AA -3′ Reverse 5′-AAA GGT GTA ACT GCA CAG GG-3′

## Data Availability

No data were used to support this study.
